# Lower Limb Joint Nursing and Rehabilitation System Based on Intelligent Medical Treatment

**DOI:** 10.1155/2021/6646977

**Published:** 2021-02-09

**Authors:** Tianjun Geng, Xiaoqian Jia, Yanli Guo

**Affiliations:** Department of Joint Surgery, The Fourth People's Hospital of Jinan, Jinan 250031, Shandong, China

## Abstract

With the aggravation of the problem of aging population, all kinds of lower limb paralysis caused by various diseases occur frequently. People's demand for lower limb nursing and rehabilitation treatment is growing. In this paper, combined with intelligent medical technology and lower limb kinematics model, this paper proposes to build a lower limb joint nursing and rehabilitation system based on intelligent medical treatment. It is expected that, through the following limb joint rehabilitation robot as the main rehabilitation means, a smart nursing rehabilitation system which can quickly respond to users and realize remote rehabilitation nursing can be designed. First of all, it is clear that the main body of the lower limb joint rehabilitation system consists of the robot body and the state display system. Then, the sensor, amplifier, and data acquisition card are set in the data acquisition system, and the plantar balance force is detected using a FlexiForce film pressure sensor. The final control system mainly includes the main control module program and the lower limb action recognition program. The motor control software adopts PID regulation method, and the lower limb action recognition adopts SVM one-to-one classification method. After the construction of lower limb joint nursing and rehabilitation system, the accuracy rate of action recognition and classification was tested. In the third experiment, the accuracy of all the movements was 100%. Then, the joint displacement and angle changes of the experimenter assisted by the system were analyzed. The experimenter's knee joint and hip joint show a normal walking state, and the joint angle changes tend to be normal. Ten out of 55 rehabilitation system users were randomly selected for interview survey. The total scores of operation convenience, wearing comfort, intensity suitability, and movement science of the system were 90, 83, 84, and 91, respectively. This shows that the rehabilitation action designed by the system is scientific and easy to operate and can be put into use in rehabilitation training after improving the wearing comfort.

## 1. Introduction

### 1.1. Background Significance

At present, Internet of things technology is developing rapidly [1]. The proposal of “Internet plus” provides a favorable opportunity for solving problems in all fields of society. For a long time, there are many problems in medical rehabilitation treatment, such as long time span, heavy work, and patients' mobility, especially for patients who need lower limb rehabilitation nursing [2]. In the increasingly aging modern society, various diseases such as stroke, joint injury, and hemiplegia cause more and more lower limb paralysis, also increasing people's rehabilitation needs [3]. How to meet the growing demand for rehabilitation so that patients can be treated in time and get adequate and scientific rehabilitation nursing is the purpose of this paper. Therefore, based on the intelligent medical technology and lower limb kinematics model, this paper proposes a lower limb joint nursing and rehabilitation system. The purpose of this paper is to design a kind of lower limb joint rehabilitation robot to carry out the simulation training of lower limb care and rehabilitation, and construct a kind of lower limb joint rehabilitation robot as the main rehabilitation means, which can quickly respond to the needs of users and realize the intelligent nursing and rehabilitation system of remote home rehabilitation nursing.

### 1.2. Related Work

Intelligent medical treatment is a new technology form in modern society [4]. It is the product of the combination of science, technology, and medicine. It can provide people with medical services beyond the limitation of time and space. It is of positive significance to improve people's living standards and improve the treatment efficiency of medical institutions. As early as the birth of smart medicine, people have a preliminary exploration on it. Lv et al. proposed a rehabilitation training scheme for upper limbs of hemiplegic patients based on wearable device HTC VIVE [5] and proposed a task-oriented rehabilitation training system design and implementation. Their experiments show that the training task effectively promotes the enthusiasm of patients to participate in rehabilitation training, which can timely feed back the movement track record of limb movement and can also meet the requirements of rehabilitation training [6]. According to Su et al., the electric intelligent lower limb prosthesis can drive the knee and ankle joints, so that the femoral amputee can make a seamless transition between motion states with the help of intention recognition system. They used machine learning technology to explore the mapping relationship between the motion state of the healthy leg and the movement intention of the cut-off before the prosthesis transition [7, 8]. Based on the data collected by a single IMU located on the lower leg, Bonnet et al. studied the possibility of estimating 3D lower limb joint kinematics in five popular hip and knee rehabilitation exercises [9]. Their research provides a reference for lower limb joint rehabilitation training, but during the experiment, the method of analyzing the data obtained from the experiment was not novel and efficient enough, and the research took a lot of time and cost.

Liu and others pointed out that a key problem of exoskeleton control is to model and predict the wearer's gait trajectory. In this regard, they proposed a depth spatiotemporal model (DSTM) for generating knee joint trajectories of lower extremity exoskeletons. Their experimental results show that, compared with other normal gaits, the energy consumption of subjects in the new recovery gait mode is less, which means that the new recovery gait is more suitable for subjects [10]. Rifai et al. proposed a bounded control strategy for knee exoskeleton, which can ensure knee flexion and extension in the process of assistance and rehabilitation. The control law proposed by them is based on nested saturation, and its main advantage is to avoid the saturation of the actuator, so as to ensure and enhance the safety of the wearer [11]. In addition, Wang et al. believe that most stroke patients have obstacles in lower limb movement, which has caused great inconvenience to their lives. Therefore, timely and effective rehabilitation training is the key to restoring the motor function of lower limbs. Therefore, they designed a lower limb rehabilitation training system based on virtual scene. The system realizes the lower limb rehabilitation training and evaluation combined with virtual reality technology, collects and processes the plantar pressure data, controls the virtual elements in the virtual scene, and displays the training time, score, and maximum and average value of plantar pressure in the training process [12, 13]. The virtual scene treatment they studied is highly interesting, which can effectively improve patients' enthusiasm for rehabilitation training and help doctors to make targeted rehabilitation plans. In this paper, the design of rehabilitation movement is provided for reference, so that the rehabilitation process does not seem so boring.

### 1.3. Innovative Points in This Paper

In order to meet the growing demand for rehabilitation, patients with lower limb injury can seek medical treatment in time and get adequate and scientific rehabilitation nursing. On the basis of intelligent medical technology and lower limb kinematics model, this paper puts forward the nursing and rehabilitation system of lower limb joints. The innovation points of this paper are as follows: (1) the nursing and rehabilitation system of lower limb joint is created, and the main body of the system includes robot body and state display system. A FlexiForce membrane pressure sensor is used to detect the plantar balance force and collect relevant data. The system is controlled by the main control module program and the lower limb action recognition program. (2) Relevant tests on the system show that the recognition and classification accuracy of lower limb movements are relatively high, the displacement and angle changes of joints are also in line with the standard of normal human walking, the motion design is scientific, and the operation is very simple.

## 2. Intelligent Medical Treatment and Rehabilitation Treatment of Lower Limb Joint

### 2.1. Smart Medical System

#### 2.1.1. Overall Demand of Smart Medicine

The main purpose of an intelligent medical system is to realize remote transmission of physiological signals detected by portable terminal, and real-time storage and analysis, so as to provide convenient intelligent medical services for users [14]. Monitoring the physiological information of users anytime and anywhere is the basic requirement of an intelligent medical system. Some chronic diseases need long-term stable monitoring to prevent the emergence of sudden symptoms without timely assistance, which is of great significance for some elderly patients with more difficult action.

Based on modern wireless communication and portable device technology, intelligent medical care needs to meet the requirements of continuous real-time collection of user physiological information [15]. Generally, the collected physiological information includes body temperature, pulse, respiration, and ECG signals [16]. The body temperature signal can reflect whether the user has inflammation or abnormal blood circulation. Respiratory signal is also very beneficial to the detection of human health, which can be used for early diagnosis of many diseases. It is very important that ECG and pulse signals can accurately reflect the running state of the heart.

The intelligent medical system is divided into three functional modules: portable terminal, information transmission and data storage module, and intelligent medical processing module [17]. The portable terminal is responsible for collecting physiological signals of human body. The information transmission and data storage module is responsible for transmitting and storing the physiological signals collected by the terminal. If necessary, the main video transmission function can be turned on to realize the health monitoring of human body. The intelligent medical processing function module mainly displays the collected physiological signals in real time and transmits them to the diagnostic doctors.

#### 2.1.2. Wireless Transmission Technology of Intelligent Medical Treatment

Wireless transmission is an important technology of intelligent medical systems, which affects the transmission of physiological signals. At present, Bluetooth, Wi-Fi, infrared technology, and ZigBee technology are commonly used in smart medical systems.

Bluetooth technology and infrared technology are only suitable for short-distance transmission [18, 19]. Bluetooth technology can realize the data exchange between fixed devices and mobile devices and has the advantages of low power consumption and low cost. However, there is no unified standard for Bluetooth technology, which may lead to incompatibility and cannot be easily extended. The point-to-point straight-line transmission of infrared technology has the advantages of convenient connection and high transmission efficiency, but its diffraction ability is poor and cannot pass through obstacles.

Wi-Fi technology has a relatively large coverage, fast transmission rate, and simple operation, but its security performance is poor with easy disclosure of user information and high transmission power consumption. ZigBee technology has a unified standard, although the transmission rate is low, but the power consumption is also greatly reduced. When the main node of the equipment is distributed network, its transmission distance can also be expanded to several kilometers.

#### 2.1.3. Application of Intelligent Medical Treatment

Smart medical systems can be generally divided into three types: smart hospital system, regional health system, and family health system, which are mainly used in telemedicine, mobile nursing, decision support, medical material management, drug management, and medical information management [20].

Telemedicine can help solve the problems of uneven allocation of medical infrastructure resources and unbalanced regional development. Telemedicine transcends the regional limitations and realizes remote cooperation, which is conducive to the sharing and utilization of medical resources. Mobile nursing is based on wireless communication and radio frequency identification technology to realize data transmission between terminals, facilitate information exchange between doctors and patients, quickly understand and master patient information, and improve the work efficiency of medical staff.

Decision support uses data mining technology to mine and analyze medical data, so as to extract useful information to assist the medical process and improve the level and accuracy of intelligence. Medical materials management uses electronic tags and radio frequency identification technology to accurately classify and search medical equipment, which improves the management efficiency of medical materials, and can also be used for the treatment of medical waste to ensure its legitimacy.

Intelligent drug management can accurately grasp the use and inventory information of drugs, formulate a reasonable procurement plan, and improve the efficiency of drug management. Medical information management uses cloud storage technology for distributed storage of medical data, which reduces the storage cost of medical data, promotes the sharing of medical data, and is conducive to the cooperation between medical institutions.

### 2.2. Kinematic Model of Human Lower Limbs

#### 2.2.1. Structure of Human Lower Limbs

The human body's moving organs can passively bear and transmit external forces and carry out movement commands to complete various human movements. Human lower limbs are composed of bones, joints, and skeletal muscles, which constitute a complete biological movement chain [21]. If the human body wants to exercise, none of the three is indispensable. Bone is the basis of this biological chain of motion, which acts as a load-bearing and lever. The joint is the hinge, and the muscle contraction is the provider of torque, which drives the skeleton to move with the joint as the support point.

Bone is the most solid structure in human body, which plays a mechanical role in human movement. The bones of the whole body are linked together to form the scaffold of the human body. Of the 206 bones in the human body, 62 are lower limb bones, accounting for about 30% of all bones [22]. The lower limb bone includes lower limb bone and free lower limb bone. The left and right sides of the hip constitute the lower limb bone, and the remaining femur, patella, tibia, and foot constitute the free lower limb bone [23].

#### 2.2.2. Movement Mechanism of Human Lower Limbs

The movement of human lower limbs mainly depends on the hip joint, knee joint, and ankle joint. The hip joint transfers the weight of the body to the lower limbs and can complete some movements in the range of flexion and extension. In the hip joint, the main body weight bearing is the femoral head. If the femoral head appears abnormal or shows pathological changes, it will lead to hip joint pain, and the joint activity and daily walking ability will be affected [24]. The knee joint is the hinge of lower limb movement, located in the middle area of lower limb. Knee joint is the most complex joint, which helps the human body to complete the posture of standing, walking, running, and jumping in daily life. The knee has a special meniscus, so it can not only stretch and bend, but also do a certain range of rotation [25]. Ankle joint mainly bears the function of load-bearing, which is an important part of the contact between human body and the ground to ensure the stable gait of lower limbs.

Walking and standing are the most basic and important two simple actions in daily life, which are the basis for completing other complex movements. Walking is the translational motion of human body and the cycle of gait cycle. Gait cycle can be divided into different gait phases according to posture changes, and gait phases are generally divided into support phase and swing phase [26]. Standing up belongs to the transformation movement, indicating that the human body is separated from the rest state and ready for other actions. The process of standing up can be divided into forward leaning stage, accelerated extension stage, and stable stage.

#### 2.2.3. Method of Establishing Dynamic Model of Human Lower Limbs

The Denavit–Hartenberg modeling method establishes a coordinate system on each connecting rod in the system and uses a 4 × 4 homogeneous transformation matrix to express the relative position of and relationship between the coordinates [27]. The position coordinates of the center of mass of the connecting rod are shown below:

(1) $$\begin{array}{c} x=\sum_{j=1}^{i=1}\left(c_{i}l_{i}\sin\;\theta_{j}\right)+d_{i}\sin\;\theta_{i}+x_{e}, \end{array}$$

(2) $$\begin{array}{c} y=\sum_{j=1}^{i=1}\left(c_{i}l_{i}\cos\;\theta_{j}\right)+d_{i}\cos\;\theta_{i}+x_{e}, \end{array}$$

where *c*_*j*_ is the member parameter; *l*_*i*_, *θ*_*i*_ are the length of the *i* member and its angle with the vertical direction; and *d*_*i*_ is the distance between the mass center of the member and the joint.

The general theorem of dynamics is derived from Newton's differential equations of motion. They include momentum theorem, momentum moment theorem, and kinetic energy theorem. Their expressions are as follows:

(3) $$\begin{array}{c} F_{c}=mv-mv_{0}, \end{array}$$

(4) $$\begin{array}{c} F=mv_{a}, \end{array}$$

(5) $$\begin{array}{c} W=\frac{1}{2}mv^{2}-\frac{1}{2}mv_{0}^{2}, \end{array}$$

where *F*, *F*_*c*_ represent the resultant external force and impulse of the object respectively; *v*, *v*_0_, *v*_*a*_ represent the velocity at the end of the body, the velocity at the initial moment, and the acceleration of the object, respectively; and *m*, *W* represent the mass of the object and the work done by the combined external force.

The focus of Lagrange modeling is to understand how the motion equation controls the robot, and use the torque equation to describe the dynamic characteristics of the robot. The equation is

(6) $$\begin{array}{c} \gamma =\frac{d}{d_{t}}\left(\frac{\partial l}{\partial v}\right)-\frac{\partial l}{\partial z}, \end{array}$$

where *γ*, *l* represent the torque and Lagrangian quantity of the system respectively, and *v*, *z* represent the generalized velocity and generalized coordinate of the system, respectively. Lagrange equation is

(7) $$\begin{array}{c} l=E-S. \end{array}$$

*E*, *S* denote kinetic energy and potential energy, respectively. The robot is affected by gravity and torque, so the part of inertial force can be placed on one side of the equation of inertial force for mechanical analysis of inertial force, as shown below:

(8) $$\begin{array}{c} \frac{\text{d}}{{\text{d}}_{t}}\left(\frac{\partial E}{\partial v}\right)-\frac{\partial E}{\partial z}=\gamma -G;G=\frac{\partial S}{\partial z}, \end{array}$$

where *G* is the gravity of the object. Transform formula (8) into

(9) $$\begin{array}{c} M\left(z\right)v_{a}+V\left(z,v\right)=\gamma -G\left(z\right). \end{array}$$

According to formula (10), the force on the object is solved.

(10) $$\begin{array}{c} \frac{\text{d}}{{\text{d}}_{t}}\left(\frac{\partial E}{\partial v}\right)-\frac{\partial E}{\partial z}=\gamma -G,\\ E=\frac{1}{2}v^{T}M\left(z\right)v. \end{array}$$

Therefore, the form of the mass matrix is derived as shown in

(11) $$\begin{array}{c} M\left(z\right)v_{a}+V\left(z,v\right)+G\left(z\right)=\gamma . \end{array}$$

Newton Euler method decomposes the general motion of a rigid body into translation and rotation around a point. The translation is solved by Newton's law, and the rotation is solved by Euler equation:

(12) $$\begin{array}{c} f=jv_{a}, \end{array}$$

(13) $$\begin{array}{c} p\varepsilon +\varepsilon \times \left(p\varepsilon \right)=\tau , \end{array}$$

where *j*, *p* represent the mass and moment of inertia of the rigid body, respectively, and *v*_*a*_, *ε* represent the acceleration and angular velocity of the rigid body, respectively.

Kane modeling method introduces the concepts of partial velocity and angular velocity. The specific steps are as follows: Firstly, the linear expression of generalized velocity is established:

(14) $$\begin{array}{c} U_{r}=\sum_{s=1}^{n}Z_{rs}v_{s}+T_{r},\;r=1,2,\ldots ,n. \end{array}$$

Then, the concepts of bias velocity and angular velocity are introduced:

(15) $$\begin{array}{c} \overset{⟶}{v}=\sum_{r=1}^{n}{\overset{⟶}{v}}_{r}U_{r}+{\overset{⟶}{v}}_{t}, \end{array}$$

(16) $$\begin{array}{c} \overset{⟶}{\varepsilon }=\sum_{r=1}^{n}{\overset{⟶}{\varepsilon }}_{r}U_{r}+{\overset{⟶}{\varepsilon }}_{t}. \end{array}$$

The generalized active force *K* and the generalized inertial force *K*′ are constructed. Assuming that any particle has an active force *F*, the expressions of the generalized active force and the inertial force are shown, respectively, as follows:

(17) $$\begin{array}{c} K=\sum_{i=1}^{n}F\cdot {\overset{⟶}{v}}_{i},\;i=1,2,\ldots ,n, \end{array}$$

(18) $$\begin{array}{c} K^{\prime }=\sum_{i=1}^{n}F^{\prime }\cdot {\overset{⟶}{v}}_{i}=\sum_{i=1}^{n}\left(-m_{i}a_{i}\right)\cdot {\overset{⟶}{v}}_{i}. \end{array}$$

Finally, Kane equation is derived according to the above formula, as follows:

(19) $$\begin{array}{c} K_{i}+K_{i}^{\prime }=0. \end{array}$$

### 2.3. Rehabilitation Robot

#### 2.3.1. Lower Limb Rehabilitation Training Mode

The purpose of lower limb rehabilitation training is to enable the abnormal lower limbs to exercise properly and effectively, promote the healing of damaged joint tissue, enhance the muscle strength of lower limbs, improve the toughness of tendons and ligaments, and improve the mobility, stability, and coordination of joints, so as to gradually recover [27, 28].

Therefore, rehabilitation training can play a great role in the recovery of lower limb function. However, different training methods need to be developed according to different degrees of damage. Rehabilitation training can be divided into passive, assisted, active, and impedance modes [29]. Passive mode is suitable for patients with complete loss of motor ability. Gait movement is completely driven by instruments, and the limbs are passively extended and reciprocated with the help of external force. Assistance mode is suitable for patients with slight recovery of movement ability but insufficient strength. The equipment provides assistance to enable people to complete gait movement. The first mock exam is to help the body remove the weight of the lower extremities and provide protection and data feedback for the patients' movement. Impedance mode is used for further training by rehabilitation patients. The equipment not only does not provide assistance, but also provides resistance to promote muscle contraction and achieve better gait movement.

The period of rehabilitation training can be divided into four stages: preparation period, recovery period, rehabilitation evaluation period, and functional rehabilitation period [30]. In these four stages, passive, assisted, active, and impedance modes can be used for functional training. At the same time, when using the rehabilitation training mode, it is necessary to choose different sports environment. For example, in passive and booster modes, it is better to choose a flat training platform with low difficulty. In active and impedance mode, the slope and step environment with higher difficulty can be selected.

#### 2.3.2. Recognition and Classification of Lower Limb Movements

Generally speaking, the most basic lower limb movements that rehabilitation robots need to recognize are forward, backward, left turn, and right turn. These four movements correspond to the flexion and extension of the knee joint and the internal and external rotation of the hip joint. For the classification of human lower limb movements, intelligent methods such as Bayesian classifier, multilayer neural network, and support vector machine (SVM) are commonly used [31].

Bayesian classifier uses fewer parameters; even some missing data will not affect the classification results; the operation is relatively simple. However, prior probability needs to be calculated before classification, so the accuracy of classification results is not high. Multilayer neural network has good self-learning ability and accurate classification ability, but the algorithm is complex and takes a long time to learn.

The complexity of SVM algorithm has little relationship with the dimension of feature samples, so it has good robustness. The core idea is that when the unknown feature vector is linearly separable, the classifier is used to find the optimal plane for classification; when the unknown feature vector is linearly separable, SVM projects it into a high-dimensional space and converts it into a linearly separable one.

#### 2.3.3. Control Strategy of Rehabilitation Robot

The control strategy of rehabilitation robot needs to be adjusted according to different training modes. In the passive training mode, the patient passively accepts the robot's power to move. In order to ensure the stability of patients' rehabilitation movement and make them receive treatment easily, the control strategy should mainly control the motor speed, limit the output torque of the drive motor, and move according to the constant speed.

In the assisted training and active training mode, patients have certain ability to autonomously move, and the control strategy of rehabilitation robot is mainly speed control. After setting the ideal speed of the motor, the patient's main motion drives the robot, but the patient's muscle strength is weak, so the motor can accelerate to reach the set ideal speed.

In impedance mode, patients need to overcome resistance for rehabilitation training. The control strategy of rehabilitation robot can control the output torque and running speed of motor. Set the motor speed to zero, and then determine the size of the motion resistance according to the torque range [30]. Adjust the resistance according to the patient's condition to help the patient improve the exercise ability.

## 3. Experiments on Construction of the Intelligent Nursing Rehabilitation System

### 3.1. Overall System Design Scheme

#### 3.1.1. Design Requirements

In this paper, the main purpose of the design of lower limb joint rehabilitation system is to help patients with lower limb dyskinesia to carry out gait rehabilitation training, by driving ankle joint to carry out gait training according to the track, driving knee joint and hip joint to move, so as to restore the walking function of lower limbs. In addition to practicability, which needs to be considered first, some technical requirements should also be considered.

The trajectory of rehabilitation robot under this system should be similar to that of normal people, which is suitable for most patients. The maximum bearing capacity of the system must be higher than 75 kg, and the actual floor space should not be too large. The height of the seat can be adjusted to meet the needs of patients of different body types. Because some of the patients may be elderly and unfamiliar with electronic products, the operation must be simplified.

#### 3.1.2. Components of the Subject

The main body of the lower limb joint rehabilitation system consists of robot body and state display system.

As shown in Figure 1, the main body of the robot mainly includes left and right foot pedal mechanism, big and small leg mechanism, and power transmission mechanism, while the state display system is mainly used to realize human-computer interaction. Patients can choose the rehabilitation training mode on the PC and adjust the movement speed.

### 3.2. Data Acquisition System

The lower limb joint rehabilitation system needs to collect the relevant data of patients in real time to provide data reference for doctors. One part of the data used for diagnosis and the next step of rehabilitation training program is collected by sensors, and the other part is obtained by reasonable analysis based on the collected data.

In the data acquisition system, the sensor is responsible for converting non-electrical physical signals into analog signals, so it is necessary to have strong anti-interference. The amplifier is responsible for amplifying and processing the voltage of the signal returned by the sensor, so it needs the characteristics of high input impedance and high common mode rejection ratio. After the output of the sensor and amplifier, the data acquisition signal must be discretized and digitized to be recognized by the computer. The detection of plantar balance force is realized by plantar pressure sensor, and the changes of plantar pressure during the movement of patients are monitored in real time, because the installation of the plantar pressure sensor cannot interfere with the movement of the patient and must have a good time delay and repeatability. A FlexiForce thin-film pressure sensor was selected for this paper.

### 3.3. Control System

The control system of the lower limb joint rehabilitation system constructed in this paper mainly includes the main control module program and the lower limb movement recognition program. The main control module includes data acquisition system, handle module, Bluetooth module, and motor control module. The data acquisition system uses sensors to collect data, preprocess it, and extract characteristic values. The handle module can ensure the stability of the system. In addition to realizing human-computer interaction on PC, patients can also control the system through the handle, which makes the operation easier. In this paper, Bluetooth module is used for communication. Bluetooth mode can realize efficient and safe short-distance transmission, which is suitable for this system. The motor control software uses PID regulation method to compare the input data with the reference value and feed back the comparison results in real time, which can improve the accuracy and stability of the system.

The lower limb movements were identified and classified by SVM one-to-one classification method. First, all the action samples should be put into the classifier at the top level; the voting results of each classifier should be put into the classifier at the next level, until the classifier at the bottom gives the classification results of the actions; and finally the data should be saved.

## 4. Discussion on the Performance of the Intelligent Nursing Rehabilitation System

### 4.1. Classification Accuracy of the System

The subjects and the lower limb joint rehabilitation system were tested for five times of recognition and classification of lower limb movements, including forward, backward, left turn, and right turn. In each test, the experimenter randomly made one of the actions, 50 times each, with a total of 200 times. The results are as follows.

As shown in Table 1, in the five experimental tests, the recognition and classification of forward and backward movements by the lower limb joint rehabilitation system were more accurate, and only two errors occurred. However, the accuracy of recognition and classification of left turn and right turn is poor and only once is correct.

As shown in Figure 2, in the third experimental test, the lower limb joint rehabilitation system accurately identified and classified all the lower limb movements made by the experimenter. In the first and fourth experiments, there are some errors in the recognition and classification of the four actions. The results are as follows.

As shown in Table 2, in the third test, the accuracy of the lower limb joint rehabilitation system in identifying and classifying all the movements made by the subjects was up to 100%. The experiment with the lowest accuracy was the first experiment, in which the system incorrectly identified and classified three left-turn actions as right-turn actions.

As shown in Figure 3, in the five recognition and classification tests for four actions, the number of times with 100% accuracy accounted for 45% of the total number of times, in which the forward and backward actions accounted for 34%, while the left-turn and right-turn actions accounted for 11%. This shows that the system has a high accuracy in the recognition of forward and backward movements, with slightly inferior accuracy in the recognition of left-turn and right-turn movements, which needs to be improved in the later experiments.

### 4.2. Joint Motion State

#### 4.2.1. Changes of Joint Displacement

In the experiment, 50 time points were selected to record the three-dimensional coordinates of knee joint and hip joint at each time point, and the time displacement coordinate curve within 3 seconds was simulated by MATLAB software. The *x*-axis represents the forward direction, and the *y*-axis represents the direction of the human body standing.

As shown in Figure 4, the changes of knee joint in the front and back directions of human walking show linear motion characteristics between 0.5 s and 2.5 s; the height of knee joint in the upper and lower direction of human walking reaches the maximum value at 1.2 s and then gradually decreases; the knee joint shows a left-right shaking motion state in the left and right directions of human walking.

As shown in Figure 5, the changes of the hip joint in the front and back directions of human walking are similar to those of the knee joint and also tend to be in a straight line; the changes of the hip joint in the up and down directions of human walking present the sine curve characteristics of the right foot falling after stepping out; and the hip joint presents the movement state of slight left and right shaking in the left and right directions of human walking. This shows that with the help of lower limb joint rehabilitation robot, the experimenter's knee joint and hip joint present normal gait state.

#### 4.2.2. Changes in Joint Angle

The angle changes of knee joint and hip joint of the experimenters in the use of lower limb joint rehabilitation robot were statistically analyzed. The angle changes of knee joint and hip joint during walking gait cycle are as follows.

As shown in Table 3, when the experimenter walks in a gait cycle with the assistance of a lower limb joint rehabilitation robot, the maximum angle of the knee joint can be bent by 71.7 degrees, which occurs when 80% of the gait cycle is completed. The maximum value of 90.9% of the hip flexion angle can be achieved at this gait cycle. Drawing the change as a curve, we can clearly see the law of its change.

As shown in Figure 6, the knee joint will also have a weak curvature value in the normal walking process, so the trough of the knee joint angle change curve is not 0. The hip angle curve reaches the trough at 50% of the gait cycle and reaches the peak when the human leg is lifted. This is similar to the change of joint angle in the process of walking in healthy state, which indicates that, with the help of lower limb joint rehabilitation robot, the change of joint angle tends to normal value.

### 4.3. Trial Feedback Results

55 patients with lower limb dyskinesia were invited to try out the lower limb joint rehabilitation robot system developed in this paper. The age and course distribution of the 55 participants were as follows.

As shown in Table 4, among the 55 participants, the number of people aged 46–55 and over 56 is the largest, with 16 people in each group accounting for 29.1% of the total. The number of patients with 6–12 months and 12–24 months is the largest, with each accounting for 29.1% of the total number.

As shown in Figure 7, among the participants under the age of 35, the number of patients with disease duration of less than 6 months was the largest, being 4 people. Among the 35–45-year-old participants, the number of patients with 6–12 months of disease duration was the largest, being 6. Among the 46–55-year-old participants, the number of patients with 12–24 months of disease was the greatest, being 6. Among those who were older than 56 years old, the number of patients with a course of disease over 24 months was the greatest, being 6 people. Therefore, the distribution of age and course of disease of the experiencer reflects such a rule that the course of disease of the younger is shorter, and the course of disease of the older is longer.

Ten randomly selected from 55 experiencers were interviewed and investigated. Each experiencer was asked to rate the system for ease of operation, comfort of wearing, suitability of intensity, and scientificity of action. The score is an integer between 0 and 10. The higher the score is, the better the performance will be. The scores of 10 participants were as follows:

As shown in Table 5, the 10 experiencers gave scores of 90, 83, 84, and 91 points, respectively, to the ease of operation, comfort of wearing, strength suitability, and scientificity of action of the system. Among them, the highest score is that of the scientific movement of the system, while the lowest score is that of the comfort of wearing. This shows that the rehabilitation movement of the system is scientific, but the related equipment is not comfortable enough.

As shown in Figure 8, the total score of experiment 3 on the system was the highest (37 points); the total score of experiment 8 on the system was the lowest (32 points). The scores of each index of the system by 10 participants were 7 or above, and the distribution of each score in 7–10 was statistically analyzed.

As shown in Figure 9, there is only one score with 7 points; there are 15 scores with 8 points, among which the intensity fitness index is the highest, 6; there are 19 scores with 9 points, of which the index of easy operation is the highest, 6; there are 5 scores with 10 points, and the index of scientific action equals 3. This shows that the score is mainly concentrated in 8 and 9 points, and everyone's satisfaction with the system is high.

From Figure 10, we can see that the left picture shows the dislocation of knee joint and patella caused by exercise. We have implemented the lower limb rehabilitation training scheme designed in this paper and carried out normal nursing. The patient has gradually recovered. The normal rehabilitation picture is shown in the right picture. The nursing rehabilitation system training designed in this paper can play a great role in the recovery of lower limb function; it can especially promote the healing of damaged joint tissue, enhance lower limb muscle strength, improve the toughness of tendons and ligaments, and improve the range of motion, stability, and coordination of joints.

## 5. Conclusions

The main purpose of an intelligent medical system is to realize remote transmission of physiological signals detected by portable terminal, and real-time storage and analysis, so as to provide convenient intelligent medical services for users. Wireless transmission is an unavailable technology in intelligent medical systems, which directly affects the transmission of physiological signals. At present, the commonly used wireless transmission technologies include Bluetooth, Wi-Fi, infrared technology, and ZigBee technology. Smart medical systems can be divided into three types: smart hospital systems, regional health systems, and family health systems. They are mainly used in telemedicine, mobile nursing, decision support, medical material management, drug management, and medical information management.

Human lower limbs coordinate the skeleton, joints, and muscles to play their respective roles to realize the lower limb movement and walk under the reaction force of the external environment. The movement of human lower limbs mainly depends on the joints of hip joint, knee joint, and ankle joint. The purpose of lower limb rehabilitation training is to enable the abnormal lower limbs to exercise properly and effectively, promote the healing of the damaged joint tissue, enhance the muscle strength of the lower limb, improve the toughness of tendons and ligaments, and improve the mobility, stability, and coordination of joints, so as to gradually recover.

Based on intelligent medical technology and human lower limb movement model, this paper creates a nursing and rehabilitation system for lower limb joints, whose main components include robot main body and status display system. A FlexiForce membrane pressure sensor is used to detect the plantar balance force and collect relevant data. The system is controlled by the main control module program and the lower limb action recognition program. The results show that the recognition and classification accuracy of the system are high, the displacement and angle change of joints also meet the standard of normal human walking, and the designed movement is scientific and easy to operate, so it can be widely used after improving comfort.

## Figures and Tables

**Figure 1:** Main structure of lower limb joint rehabilitation system.

**Figure 2:** Distribution of system identification and classification results.

**Figure 3:** Distribution of recognition and classification accuracy of the system.

**Figure 4:** Three-dimensional curved surface of knee joint displacement.

**Figure 5:** Three-dimensional curved surface of hip joint displacement.

**Figure 6:** Variation curve of joint angle in gait cycle.

**Figure 7:** Distribution of age and course of disease of participants.

**Figure 8:** Score difference of the system.

**Figure 9:** Distribution of system scores.

**Figure 10:** Nursing and rehabilitation of patellar dislocation of knee joint.

**Table 1:** Classification results of system identification.

Times	Forward	Backward	Left	Right	Total
1	49	51	47	53	200
2	50	50	48	52	200
3	50	50	50	50	200
4	51	49	52	48	200
5	50	50	51	49	200

**Table 2:** Accuracy of system identification and classification.

Times	Forward (%)	Backward (%)	Left (%)	Right (%)
1	98	98	94	94
2	100	100	96	96
3	100	100	100	100
4	98	98	96	96
5	100	100	98	98

**Table 3:** Joint angles in gait cycle.

Gait (%)	Knee angle (°)	Hip angle (°)
10	26.3 ± 0.23	35.4 ± 0.31
20	30.1 ± 0.28	20.8 ± 0.22
30	21.8 ± 0.2	11.1 ± 0.14
40	18.4 ± 0.17	−1.5 ± 0.04
50	19.5 ± 0.15	−9.8 ± 0.13
60	38.7 ± 0.26	0.4 ± 0.05
70	65.3 ± 0.33	21.5 ± 0.21
80	71.7 ± 0.46	36.2 ± 0.28
90	26.9 ± 0.26	36.9 ± 0.33
100	15.6 ± 0.19	34.7 ± 0.29

**Table 4:** Age and course of disease of participants.

Age	<6 months	6–12 months	12–24 months	>24 months	Total
<35	4	3	2	1	10
35–45	2	6	3	2	13
46–55	2	4	6	4	16
>56	2	3	5	6	16
Total	10	16	16	13	55

**Table 5:** System score results.

Index	Simplicity	Comfort	Suitability	Scientificity
1	9	8	8	9
2	8	9	8	10
3	9	9	9	10
4	9	8	9	9
5	10	8	8	9
6	9	8	8	8
7	9	9	8	10
8	8	7	9	8
9	10	9	8	9
10	9	8	9	9
Total	90	83	84	91

## Data Availability

No data were used to support this study.
